# Identification of Key MicroRNAs and Genes between Colorectal Adenoma and Colorectal Cancer via Deep Learning on GEO Databases and Bioinformatics

**DOI:** 10.1155/2023/6457152

**Published:** 2023-02-05

**Authors:** Xin Zhang, Mingxin Jin, Fengjun Liu, Hui Qu, Cheng Chen

**Affiliations:** Department of General Surgery, Qilu Hospital of Shandong University, 107 Wenhuaxi Road, Jinan 250012, Shandong, China

## Abstract

**Background:**

Deep learning techniques are gaining momentum in medical research. Colorectal adenoma (CRA) is a precancerous lesion that may develop into colorectal cancer (CRC) and its etiology and pathogenesis are unclear. This study aims to identify transcriptome differences between CRA and CRC via deep learning on Gene Expression Omnibus (GEO) databases and bioinformatics in the Chinese population.

**Methods:**

In this study, three microarray datasets from the GEO database were used to identify the differentially expressed genes (DEGs) and differentially expressed miRNAs (DEMs) in CRA and CRC. The FunRich software was performed to predict the targeted mRNAs of DEMs. The targeted mRNAs were overlapped with DEGs to determine the key DEGs. Molecular mechanisms of CRA and CRC were evaluated using enrichment analysis. Cytoscape was used to construct protein–protein interaction (PPI) and miRNA–mRNA regulatory networks. We analyzed the expression of key DEMs and DEGs, their prognosis, and correlation with immune infiltration based on the Kaplan–Meier plotter, UALCAN, and TIMER databases.

**Results:**

A total of 38 DEGs are obtained after the intersection, including 11 upregulated genes and 27 downregulated genes. The DEGs were involved in the pathways, including epithelial-to-mesenchymal transition, sphingolipid metabolism, and intrinsic pathway for apoptosis. The expression of has-miR-34c (*P* = 0.036), hsa-miR-320a (*P* = 0.045), and has-miR-338 (*P* = 0.0063) was correlated with the prognosis of CRC patients. The expression levels of BCL2, PPM1L, ARHGAP44, and PRKACB in CRC tissues were significantly lower than normal tissues (*P* < 0.001), while the expression levels of TPD52L2 and WNK4 in CRC tissues were significantly higher than normal tissues (*P* < 0.01). These key genes are significantly associated with the immune infiltration of CRC.

**Conclusion:**

This preliminary study will help identify patients with CRA and early CRC and establish prevention and monitoring strategies to reduce the incidence of CRC.

## 1. Introduction

Colorectal cancer (CRC) is one of the malignant tumors with the highest morbidity worldwide [1, 2]. Despite advances in the detection and therapy of CRC in recent years, CRC has remained a major challenge in clinical practice [3]. Around 50%–70% of CRC comes from adenomatous polyps [4, 5]. CRC, also known as bowel cancer, is a type of cancer that forms from the growth of uncontrolled cells in the colon or rectum (part of the large intestine) or the appendix. Colorectal adenoma (CRA) is an epithelial tumor consisting of abnormal glands in the large intestine. The primary cause of CRC is adenomatous polyps, which progress to advanced CRA with highly heterogeneous hyperplasia, and finally to invasive carcinoma [6]. Classical adenomas are precursor lesions characterized by hyperplastic and dysplastic epithelial cells with increased malignant transformation potential [7]. Colorectal tumorigenesis is considered a multistep process in which genetic changes continue to accumulate, eventually resulting in an aggressive phenotype (adenoma–carcinoma sequence) [8]. Statistical analysis showed that the 5-year survival rate of patients with stage I CRC was over 90% and that of patients with stage IV CRC was only 10% [9]. It is important to identify the molecular markers of CRC as it is one of the most curable cancers if detected early [10].

In recent decades, advanced gene microarrays and high-throughput sequencing methods have been used to study CRC gene expression, therapeutic targets, and pathogenesis [11]. Analysis of gene expression microarray data with bioinformatics provides an effective tool for identifying previously unknown mRNAs and microRNAs (miRNAs) that may have a role in cancer pathogenesis [12]. CRC is associated with abnormal gene expression and mutations. Some markers, including TP53, KRAS, BRAF, and GNAS mutations, are the primary focus of research [13]. miRNAs are small noncoding RNAs with a length of 19–22 nucleotides, and they play an important role in cell growth, differentiation, and survival by completely or incompletely binding to target mRNAs, leading to mRNA degradation or post-transcription inhibition [14]. Studies have found that miRNAs are involved in CRC caused by inflammatory bowel disease [15]. Several driver gene mutations, as well as other molecular events, such as miRNA regulation or pre-mRNA splicing changes, have been detected during the progression from CRA to CRC [16]. There are big geographic differences in the global distribution of CRC, and the pathogenic factors may also be different [17, 18]. The transcriptome differences between CRA and CRC in the Chinese population remain unknown.

Deep learning (DL) is a representation learning method that learns multiple input data incrementally [19]. The availability of a large database of transcriptomic analyses offers unprecedented opportunities to use sophisticated DL algorithms to discover new predictive biomarkers [20]. The reduced cost of large-scale second-generation sequencing and the availability of such data through open-source databases (e.g., The Cancer Genome Atlas (TCGA) and Gene Expression Omnibus (GEO) databases) offer the possibility of building more powerful and accurate models to predict cancer progression more accurately [21]. In this study, three microarray datasets from the GEO database were used to identify differentially expressed genes (DEGs) and differentially expressed miRNAs (DEMs) between CRA and CRC tissues. The FunRich software was performed to predict the targeted mRNAs of DEMs, and then the targeted mRNAs were overlapped with DEGs to determine the key DEGs. A molecular enrichment analysis was conducted to evaluate the underlying molecular mechanisms involved in CRA and CRC. Cytoscape was used to construct protein–protein interaction (PPI) and miRNA–mRNA regulatory networks. We analyzed the expression of key DEMs and DEGs, their prognosis, and correlation with immune infiltration based on the Kaplan–Meier plotter, UALCAN, and TIMER databases. Our findings provide new insights for understanding the progress from CRA to CRC.

## 2. Materials and Methods

### 2.1. Microarray Data Information

The GEO database is a database that stores microarray, next-generation sequencing, and other high-throughput sequencing data. Using this database, we can retrieve some experimental sequencing data uploaded by some other people. The GEO (https://www.ncbi.nlm.nih.gov/geo/) database was used to download the gene expression profile datasets (GSE41657, GSE71187) and the miRNA expression profile dataset (GSE72281) [22]. Inclusion criteria are China-based datasets, paired normal mucosa, adnoma and adenocarcinoma tissues, and a sample size ≥5 for each group. GSE41657 was based on the platform of GPL6480, including 51 CRA tissues and 25 CRC tissues (Table 1). GSE71187 was also based on the platform of GPL6480, including 58 CRA tumor tissues and 47 CRC tissues. GSE72281 was based on the platform of GPL18058, including six CRA tumor tissues and six CRC tumor tissues. The GSE72281 dataset has not been published.

### 2.2. Identification of DEMs and DEGs

GEO2R (https://www.ncbi.nlm.nih.gov/geo/geo2r/), a built-in online tool of GEO, was used to compare CRC and CRA [23]. In this study, we focused on mRNAs and miRNAs that are significantly differentially expressed between CRC and CRA. Adjusted *P*-value < 0.05 and |logFC| > 1 were set as the thresholds for identifying DEGs and DEMs [24]. Adjusted *P*-value < 0.05 and |logFC| > 1 were defined as “upregulated” and adjusted *P*-value < 0.05 and |logFC| < 1 were defined as “downregulated.” The R package (“ggplot2”) was used to visualize the DEGs and DEMs. The FunRich software (version 3.0) was used to predict the miRNA targets. To obtain the hub genes, the targeted genes of downregulated miRNAs were intersected with the upregulated DEGs in GSE41657 and GSE71187 datasets, and the targeted genes of upregulated miRNAs were intersected with the downregulated DEGs in GSE41657 and GSE71187 datasets.

### 2.3. Gene Ontology (GO) and Pathway Enrichment Analysis

To investigate the biological processes (BP), cell components (CC), molecular functions (MF), and signaling pathways involved in DEGs, we used the FunRich software to perform Gene Ontology (GO) and pathway enrichment analysis. The results were considered statistically significant if *P*-value < 0.05 [25].

### 2.4. PPI Network Construction

PPI networks are composed of proteins that interact with each other to participate in various aspects of life processes such as biological signaling, regulation of gene expression, energy and material metabolism, and cell cycle regulation. The PPI among overlapping DEGs were identified via STRING database (https://string-db.org/), and the PPI network was constructed by choosing genes with the combined score ≥0.4 [26]. Cytoscape 3.8.0, an open-source tool for visualizing biomolecular interaction networks composed of proteins, genes, and other types of interaction, was used to analyze and visualize the PPI network [27].

### 2.5. Construction of the miRNA–mRNA Regulatory Network

miRNAs are endogenous, single-stranded, and noncoding regulatory small molecules that act in organisms by repressing gene expression. Each miRNA can have multiple target genes and, at the same time, a gene may be regulated by multiple miRNAs. Thus, this complex regulatory network can either regulate the expression of multiple genes through a single miRNA or finely regulate the expression of a gene through a combination of several miRNAs. The analysis of miRNA–mRNA regulatory networks allows a more accurate analysis of the interactions or regulatory mechanisms involved. The hub genes were paired with DEMs, and the miRNA–mRNA regulatory network was constructed by utilizing Cytoscape software [28].

### 2.6. miRNAs and the Prognosis of Patients with CRC

The sources of Kaplan–Meier plotter (https://kmplot.com/analysis/) include GEO, European Genome-phenome Archive, and TCGA, which can evaluate the influence of genes (mRNA, miRNA, and protein) on the survival rate of 21 cancer types [29]. The main aim of the tool is to discover and validate biomarkers of survival in cancer research based on meta-analysis. This method was used to determine whether miRNAs had prognostic value in CRC.

### 2.7. Validation of the Hub Genes via UALCAN Database

UALCAN (http://ualcan.path.uab.edu) is an interactive website whose resources are based on the level 3 RNA-seq and clinical data of 31 cancer types in the TCGA database, which is different from the GEO database [30]. UALCAN is a comprehensive, user-friendly, and interactive web resource for the analysis of cancer omics data. It is built on practical extraction and report language-common gateway interface with high quality graphics using JavaScript and cascading style sheets. UALCAN is designed to provide easy access to publicly available cancer omics data (TCGA, MET500, CPTAC, and CBTTC), allowing users to identify biomarkers or in silico validation of potential genes of interest, providing descriptions of protein coding expression profiles and patient survival information in charts and graphs. In this study, UALCAN database was used to validate the expression of hub genes.

### 2.8. Validation of the Hub Genes via TIMER Database

The TIMER web server is a comprehensive resource for the systematic analysis of immune infiltration in different types of cancer. Users can fully explore the clinical and genomic characteristics of tumors with TIMER's (https://cistrome.shinyapps.io/timer/) comprehensive analysis of immune infiltrates of different cancer types [31]. We examined the correlation of hub genes in CRA and CRC with six immune cells: B cells, CD8+ T cells, CD4+ T cells, macrophages, neutrophils, and dendritic cells [32].

## 3. Results

### 3.1. GEO-Based DEG and DEM Identification

Most studies do DL using only a single type of omics data to build models, but this study utilized multiple types of omics data, including mRNA and miRNA. In Supplementary Table S1, we provide DEGs and DEMs for the three datasets. There were 656 DEGs in the GSE41657 dataset, including 416 upregulated genes and 240 downregulated genes (Figure 1(a)). There were 1,436 DEGs in the GSE71187 dataset, including 846 upregulated genes and 590 downregulated genes (Figure 1(b)). There were 94 DEMs in GSE72281, including 44 upregulated miRNAs and 50 downregulated miRNAs (Figure 1(c)). There are 38 DEGs obtained after the intersection, including 11 upregulated genes and 27 downregulated genes (Figures 1(d) and 1(e)).

### 3.2. Functional Enrichment Analysis

As shown in Figure 2(a), DEGs associated with biological processes were mainly associated with cell communication, signal transduction, and fatty acid metabolism. DEGs in the cell component were mainly enriched in the cytoskeleton, the cyclic adenosine monophosphate-dependent protein kinase complex, and the membrane coat adaptor complex (Figure 2(b)). As a function of their molecular function, DEGs exhibited enhanced affinity for transmembrane receptor proteins, cytoskeletal protein binding, and voltage-gated ion channel activity (Figure 2(c)). Based on GO annotation, these DEGs exhibited a significant enrichment in cell communication, cytoskeleton, and transmembrane receptors. The results of biological pathway enrichment showed that the DEGs were mainly enriched in epithelial-to-mesenchymal transition, sphingolipid metabolism, and intrinsic pathway for apoptosis (Figure 2(d) and Table 2).

### 3.3. PPI Network and miRNA–mRNA Regulatory Network

When doing DL, the core genes are selected by ranking them according to their importance in biological networks, such as PPI networks [33]. As shown in Figure 3(a), 38 DEGs were filtered using the STRING database in a PPI network with 19 nodes and 32 edges. The essential miRNA–mRNA pairs were visualized by Cytoscape software. There were 16 miRNAs associated with 38 DEGs, including 11 upregulated miRNAs and five downregulated miRNAs (Figure 3(b)).

### 3.4. The Relationship between miRNA and the Prognosis of CRC Patients

Kaplan–Meier plotter was used to evaluate the prognostic values of the 16 DEMs in CRC. The overexpression of hsa-miR-34c-5p (MIMAT0000686) (*P* = 0.036) was associated with poor overall survival (OS) in patients with CRC (Figure 4(a)). However, the overexpression of hsa-miR-320a (MIMAT0000510) (*P* = 0.045), has-miR-338-3p (MIMAT0000763) (*P* = 0.0063), and has-miR-431-5p (MIMAT0001625) (*P* = 0.0065) was associated with OS in patients with CRC (Figure 4(b)–4(d)). This indicated that these miRNAs may be potential targets. Then, we validated the expression of DEGs paired with miRNAs in CRC.

### 3.5. Validation of Hub Gene Expression via UALCAN Database

There were nine hub genes paired with the hub miRNAs, including BCL2, CBFA2T3, PPM1L, ARHGAP44, PRKACB, TPD52L2, VIM, WNK4, and CD34 (Table 3). Compared with normal tissues, CRC tissues expressed significantly lower levels of BCL2 (ENSG00000171791), PPM1L (ENSG00000163590), ARHGAP44 (ENSG00000006740), and PRKACB (ENSG00000142875) (*P* < 0.001) (Figure 5(a)–5(d)). The mRNA expression levels of TPD52L2 (ENSG00000101150) and WNK4 (ENSG00000126562) in CRC tissues were significantly higher than those in normal tissues (*P* < 0.01) (Figures 5(e) and 5(f)). Three miRNAs were paired with these six genes, including hsa-miR-34c-5p, hsa-miR-320a, and hsa-miR-338-3p.

### 3.6. Relationship between the Hub Genes and Immune Infiltration

We explored the correlation of those hub genes with the immune infiltration levels in CRC using TIMER database. As shown in Figure 6, there was a significant correlation between BCL2 and PPM1L and the infiltrating levels of B cells as well as CD8+ T cells, CD4+ T cells, macrophages, neutrophils, and dendritic cells (*P* < 0.05). There was a significant correlation between ARHGAP44 levels and the infiltrating levels of B cells and CD4+ T cells (*P* < 0.05). There was a significant correlation between PRKACB and the infiltrating levels of B cells, CD8+ T cells, CD4+ T cells, macrophages, and dendritic cells (*P* < 0.05). There was a significant correlation between TPD52L2 and the infiltrating levels of B cells, CD8+ T cells, CD4+ T cells, and macrophages (*P* < 0.05). There was a significant correlation between KPNA2 and the infiltrating levels of CD8+ T cells, CD4+ T cells, neutrophils, and dendritic cells (*P* < 0.05).

## 4. Discussion

CRA is a precancerous lesion that may develop into CRC, and its etiology and pathogenesis are not yet clear [34]. Previous studies have investigated the genetic alterations in CRA and CRC samples [35]. Nevertheless, discrepant results were gained owing to different countries, platforms, and control selection. Our study discussed the transcriptome differences between CRA and CRC in the Chinese population.

In this study, we identified DEGs and DEMs associated with CRA and CRC. We identified 38 key DEGs, including 11 upregulated genes and 27 downregulated genes. According to GO annotation results, DEGs are mainly associated with cell communication, cytoskeleton, and transmembrane receptors. The results of biological pathway enrichment showed that the DEGs were mainly enriched in epithelial-to-mesenchymal transition, sphingolipid metabolism, and intrinsic pathway for apoptosis. Cancer progression as well as therapeutic resistance is influenced by the epithelial–mesenchymal transition (EMT) [36]. EMT is the process by which epithelial cells undergo a series of biochemical changes to acquire a mesenchymal phenotype. A variety of tumors exhibit drug-resistance mechanisms due to dysregulation of sphingolipid metabolism. ECHS1 induces sphingolipid-metabolism imbalance to promote CRC progression by regulating ceramide glycosylation [37]. Mitochondrial dysfunction regulates apoptosis through an intricate process controlled by complex interactions between B-cell lymphoma 2 (Bcl-2) family members and other cellular proteins [38]. In colorectal tissue, the imbalance between cell proliferation and apoptosis usually leads to tumor growth [39]. The intrinsic pathway for apoptosis responds to various types of intracellular stress, including growth factor withdrawal, DNA damage, unfolding stress in the endoplasmic reticulum, and death receptor stimulation.

The essential miRNA–mRNA pairs were constructed via Cytoscape software. Then, we identified three miRNAs (hsa-miR-34c-5p, hsa-miR-320a, and hsa-miR-338-3p) and six genes (BCL2, PPM1L, ARHGAP44, PRKACB, TPD52L2, and WNK4) based on Kaplan–Meier plotter and UALCAN database. In cancer cells, miR-34c expression decreases due to abnormal DNA methylation [40]. miR-34c plays a role of tumor suppressor in endometrial carcinoma cells by targeting E2F3 protein [41]. Using miR-320a to suppress colon cancer cells can help predict prognosis and treat cancer [42]. miRNA-338-3p could inhibit colorectal carcinoma cell invasion and migration by inhibiting smoothened expression [43]. Cell death regulator BCL2 plays an important role in controlling mitochondrial cytochrome c release and inhibiting proapoptotic genes [44]. We found low expression of BCL2 in the databases, which may be due to its different role in different cancer species. PPM1L is a likely candidate tumor suppressor gene whose downregulation can modulate colorectal tumorigenesis [45]. Rho GTPase activating protein 44 (ARHGAP44) is a Rho GAP domain-containing protein. Bioinformatics analysis showed that ARHGAP44 was less expressed in lung cancer tissues than in normal tissues and verified by quantitative real-time PCR (qRT-PCR) using patient specimens [46]. Protein kinase catalytic subunit *β* (PRKACB) is a member of the serine/threonine protein kinase family. It is a key regulatory point for cell proliferation, differentiation, and apoptosis regulation, and is closely related to cell growth, tumor proliferation, metastasis, and other physiological and pathological processes [47]. CRC patients with PRKACB downregulation have worsened OS [47]. TPD52L2 impacts proliferation, invasiveness, and apoptosis of glioblastoma cells via modulation of Wnt/*β*-catenin/snail signaling. However, its role in CRC is unclear [48]. WNK4 was identified as contributing to both cell proliferation and resistance to cisplatin treatment in medulloblastoma cells [49].

The accuracy of cancer progression prediction will greatly benefit the clinical management of cancer patients [21]. Improvements in translational biomedical research and the application of advanced statistical analysis and machine learning methods are driving the improvement of cancer progression prediction [21]. Due to the limited clinical hair information of the three GEO databases included in this study, it is currently not possible to continue to construct predictive models for progression from CRA to CRC based on the six core DEGs and three DEMs obtained. We will do core gene-based model prediction and validation in more datasets or real-world samples in the future.

The results of this study provide useful information for CRA and CRC. However, this study has some limitations, such as the number of GEO datasets used in this research is relatively small, thus more datasets should be used in future research to identify DEMs and DEGs. Besides, molecular experiments are required to confirm these results.

## 5. Conclusion

There were 38 DEGs between CRC and CRA. The DEGs were involved in the pathways, including epithelial-to-mesenchymal transition, sphingolipid metabolism, and intrinsic pathway for apoptosis. The progression of CRA to CRC may be influenced by three key DEMs (hsa-miR-34c-5p, hsa-miR-320a, and hsa-miR-338-3p) and six key DEGs (BCL2, PPM1L, ARHGAP44, PRKACB, TPD52L2, and WNK4). These key genes are significantly associated with the immune infiltration of CRC. This preliminary study will help identify patients with CRA and early CRC and establish prevention and monitoring strategies to reduce the incidence of CRC.

## Figures and Tables

**Figure 1:** Volcano plot and Venn diagrams of the DEGs and DEMs in several GEO datasets: (a) the DEGs in GSE41657 dataset; (b) the DEGs in GSE71187 dataset; (c) the DEMs in GSE72281 dataset; (d) the upregulated DEGs in three datasets; (e) the downregulated DEGs in three datasets. DEGs: differentially expressed genes; DEMs, differentially expressed microRNAs.

**Figure 2:** The results of GO and pathway enrichment analysis for DEGs. The top 10 of (a) biological process, (b) cellular component, (c) molecular function, and (d) biological pathways of the DEGs. GO, Gene Ontology.

**Figure 3:** The PPI and microRNA–mRNA regulatory networks of key DEMs and DEGs: (a) the PPI network of the DEGs; (b) the microRNA–mRNA regulatory network of key DEMs and DEGs. Red indicates upregulated miRNAs and genes, and blue indicates downregulated miRNAs and genes. PPI, protein–protein interaction.

**Figure 4:** The association between key microRNAs and CRC prognosis. CRC, colorectal cancer.

**Figure 5:** The expression levels of key genes in COAD samples: (a) BCL2; (b) PPM1L; (c) ARHGAP44; (d) PRKACB; (e) TPD52L2; (f) WNK4.

**Figure 6:** Correlation between the gene expression of genes and immune cells in CRC: (a) BCL2; (b) PPM1L; (c) ARHGAP44; (d) PRKACB; (e) TPD52L2; (f) WNK4. CRC, colorectal cancer. *P* < 0.05 was considered statistically significant.

**Table 1:** Basic information of three gene microarray datasets.

Data source	Series	Platform	Sample size (CRA/CRC)
mRNA	GSE41657	GPL6480	51/25
mRNA	GSE71187	GPL6480	58/47
miRNA	GSE72281	GPL18058	6/6

CRA, colorectal adenoma; CRC, colorectal cancer.

**Table 2:** Pathway enrichment analysis of hub genes associated with CRC progression.

Biological pathway	No. of genes in the dataset	Fold enrichment	*P*-value	Genes mapped
Epithelial-to-mesenchymal transition	4	6.489	0.002928	AP1S2, ZCCHC24, VIM, SPARC
Sphingolipid metabolism	2	20.743	0.004083	PPM1L, ACER2
Intrinsic pathway for apoptosis	2	19.405	0.004657	VIM, BCL2
FGFR2c ligand binding and activation	1	150.436	0.006667	FGFR2
Asparagine degradation I	1	150.436	0.006667	ASRGL1
BH3-only proteins associate with and inactivate antiapoptotic BCL2 members	1	100.457	0.009984	BCL2
Caspase cascade in apoptosis	2	11.570	0.012733	VIM, BCL2
ATF2 transcription factor network	2	10.198	0.016201	BCL2, PPARGC1A
CREB phosphorylation through the activation of adenylate cyclase	1	60.354	0.016587	PRKACB
Activation, myristoylation of BID, and translocation to mitochondria	1	60.354	0.016587	VIM

**Table 3:** The hub DEMs and DEGs in CRA and CRC.

miRNAs	Up/down	Targeted genes	Up/down
hsa-miR-34c-5p	Upregulated	BCL2	Downregulated
hsa-miR-34c-5p	Upregulated	CBFA2T3	Downregulated
hsa-miR-34c-5p	Upregulated	PPM1L	Downregulated
hsa-miR-34c-5p	Upregulated	ARHGAP44	Downregulated
hsa-miR-34c-5p	Upregulated	PRKACB	Downregulated
hsa-miR-320a	Downregulated	TPD52L2	Upregulated
hsa-miR-320a	Downregulated	VIM	Upregulated
hsa-miR-338-3p	Downregulated	WNK4	Upregulated
hsa-miR-431-5p	Downregulated	CD34	Upregulated

CRA, colorectal adenoma; CRC, colorectal cancer.

## Data Availability

The data used to support the findings of this study are available from the corresponding author upon request.

## Supplementary Materials

Supplementary Materials Table S1: The DEGs and DEMs of GSE41657, GSE71187, and GSE72281.
